The article "Effects of uric acid on endothelial dysfunction in early chronic kidney disease and its mechanisms" was retracted in 2015. Reasons: compromised peer review; ethical violations by an institution or third party; concerns about the results or conclusions.

# Effects of uric acid on endothelial dysfunction in early chronic kidney disease and its mechanisms

**DOI:** 10.1186/2047-783X-18-26

**Published:** 2013-07-30

**Authors:** Yu Wang, Xiaorong Bao

**Affiliations:** 1 Department of Nephrology, Jinshan Hospital affiliated to Fudan University, No.1508 Longhang Road, Jinshan District, Shanghai 201508, China

**Keywords:** Early chronic kidney disease, Endothelial dysfunction, Lipid oxidation, Micro-inflammation, Oxidative stress, Uric acid

## Abstract

**Background:**

An increase in serum uric acid (UA) occurs during the early and middle stages of chronic kidney disease (CKD) and aggravates the deterioration of kidney function. This study aims to explore the relation between UA and endothelial dysfunction in early CKD and its mechanisms in a murine model.

**Methods:**

The experimental animals were randomly divided into three groups (n = 10): sham-operation group (control group), right nephrectomy only group (CKD group) and right nephrectomy with oxonic potassium group (CKD with hyperuricemia group). Furthermore, we analyzed the relation between UA and endothelial dysfunction indices in early CKD as well as its mechanisms.

**Results:**

Linear regression analysis showed that the level of serum UA had a significant positive correlation with serum endothelin-1 and the percentage of collagen I positive area, but a negative correlation with serum nitric oxide (NO) and NO/endothelin-1 ratio. In addition, the level of serum UA had significant positive correlations with serum malonaldehyde, serum C-reactive protein, serum oxidatively-modified low-density lipoprotein and serum low-density lipoprotein, but a negative correlation with serum superoxide dismutase.

**Conclusions:**

Endothelial dysfunction in the CKD group was significant and had a positive correlation with the level of serum UA. Endothelial dysfunction in early CKD with hyperuricemia is perhaps related to oxidative stress, micro-inflammation and lipid oxidation.

## Background

Since previous studies have highlighted the role of serum uric acid (UA) in coronary heart disease [1], the effect and mechanism of UA in cardiovascular disease (CVD) has aroused widespread concern. Serum UA level is not only the most significant predictor of occurrence of primary hypertension [2], but it is also associated with cardiovascular morbidity and mortality [3-5].

Chronic kidney disease (CKD) affects 10–13% of the general population. CKD patients have an extremely high risk of developing CVD compared with the general population. Patients in the early stages of CKD are more likely to convert into CVD rather than progress towards end-stage renal disease [6]; CVD is the major cause of death in patients with CKD [7]. The increase in serum UA occurs in the early and middle stages of CKD and aggravates with the deterioration of kidney function [8]. At present, no publication has demonstrated the effect and mechanism of UA in early CKD with CVD patients. Our earlier clinical study found that serum UA was increased in patients with stage 2–3 CKD and was related to CVD (e.g. left ventricular hypertrophy), indicating that hyperuricemia was associated with CVD in early CKD.

The article "Effects of uric acid on endothelial dysfunction in early chronic kidney disease and its mechanisms" was retracted in 2015. Reasons: compromised peer review; ethical violations by an institution or third party; concerns about the results or conclusions.

Endothelial dysfunction is an early occurrence in CVD. Vascular endothelial cells play an important role in cellular functions, such as modulating angiokinesis, the proliferation and migration of vascular smooth muscle cells, anti-platelet aggregation, and extracellular matrix generation. Pathological changes in blood vessels, including intima hyperplasia, lumen straightness and atherosclerosis, are a consequence of endothelial dysfunction. In the clinic, endothelial dysfunction is associated with CVD, and specifically with hypertension, coronary heart disease, thrombosis, and cardiac insufficiency [9-11]. Endothelial cells can synthesize and excrete many important substances, the serum levels of which will change in the condition of endothelial dysfunction, such as decreased nitric oxide (NO) level, increased endothelin-1 (ET-1) level, and decreased NO/ET-1 ratio [12,13]. Thus, the content of NO and ET-1 is important for evaluating the function of endothelial cells. Collagen I deposition in the artery is also related to the function of endothelial cells; endothelial cell dysfunction increases the excretion of transforming growth factor-β (TGF-β) and other substances of collagenous protein synthesis, leading to the deposition of abundant collagen I in the artery.

Endothelial cell injury is generally related to genetic factors, lifestyle, age, obesity, smoking, blood pressure (pulse pressure), heart dysfunction, fasting hyperglycemia (impaired glucose tolerance) and insulin resistance. The unique status of CKD, namely oxidative stress, micro-inflammation, and lipid oxidation [14], can also cause endothelial cell injury. At present, studies exploring the mechanisms of endothelial cell injury in CKD patients mainly focus on end-stage renal disease patients. The mechanism of UA-induced endothelial damage in early CKD is not well known.

Despite recent advances in the treatment of CKD, the disease remains an important public health challenge [15]. Traditional risk factors, such as hypertension and hypercholesterolemia, cannot explain the excess cardiovascular mortality in CKD patients. Identifying and treating risk factors of early CKD may be the best approach to prevent and delay adverse outcomes [16]. Through the establishment of early CKD animal models with elevated serum UA, we explored the relationship between UA and vascular endothelial cell damage, and further investigated the mechanisms of injury in order to elucidate intervening CVD risk factors as early as possible in CKD patients.

The article "Effects of uric acid on endothelial dysfunction in early chronic kidney disease and its mechanisms" was retracted in 2015. Reasons: compromised peer review; ethical violations by an institution or third party; concerns about the results or conclusions.

## Methods

### Reagents and antibodies

NO, superoxide dismutase (SOD), and malondialdehyde (MDA) detection kits were purchased from Nanjing KeyGEN Biotech. Co. Ltd. (Nanjing, China). Oxidatively modified low-density lipoprotein (ox-LDL), ET-1, and C-reactive protein (CRP) detection kits were purchased from ADL (Adlitteram Diagnostic Laboratories, USA). Diaminobenzidine chromogenic kit, rabbit anti-mouse collagen I polyclonal antibody, and goat anti-rabbit polyclonal antibody were purchased from Fuzhou Maixin Biotechnology Co. Ltd. (Fujian, China). Beckman CX9 biochemical analyzer and Beckman supporting reagents were purchased from Beckman Coulter (USA).

### The establishment of early CKD animal model with hyperuricemia

Thirty male Sprague-Dawley rats, weighing 187 g to 232 g and 6 to 7 weeks old, obtained from Xipuer-bikai experimental animal company (Shanghai, China), were employed in the present study. All experimental procedures were conducted in accordance with the Guiding Principles for the Care and Use of Animals in Research and Teaching, approved by the Institutional Animal Care and Use Committee of Jinshan Hospital affiliated to Fudan University, China.

The experimental animals were randomly divided into three groups (n = 10): sham-operation group (control group, Group A), right nephrectomy-only group (CKD group, Group B), and right nephrectomy with oxonic potassium group (CKD with hyperuricemia group, Group C). The rats were housed in standard plastic cages; food and water were freely available.

The experimental animals were anesthetized using an intraperitoneal injection at a dose of 5% ketamine (100 mg/kg). The surgical region was shaved and the shin was cleaned with 75% alcohol. The right kidney was exposed through a longitudinal incision under the right costal arch (proximal to the right side of the spine). For Groups B and C, the right kidney was resected. The entire procedure was performed in the sham group, but nephrectomy was not applied. After one week of normal feeding, the rats in all three groups were in good condition. The experimental group was fed with uricase inhibitor (oxonic potassium) twice a day (800 mg/kg, at 8 a.m. and 5 p.m.) by gavage. During the experiment, rats were weighed every two weeks and the administered dose was adjusted based on body weight. Unilateral nephrectomy group and the sham-operation group were fed with the same amount of saline.

The article "Effects of uric acid on endothelial dysfunction in early chronic kidney disease and its mechanisms" was retracted in 2015. Reasons: compromised peer review; ethical violations by an institution or third party; concerns about the results or conclusions.

### Sample collection and management

After ten weeks of gavage administration, rats were killed and blood samples were collected from the heart into non-heparinized tubes. The blood sera were then collected via centrifugation and stored at −70°C for detection of UA, serum creatinine (Scr), NO, ET-1, CRP, MDA, SOD, ox-LDL, and LDL. For light microscopic examination, left kidney tissues from each group were fixed with 10% formalin, stored at 4°C for 14 to 16 hours, and then embedded with paraffin. After routine processing, paraffin sections of each tissue were cut into 4-μm thickness and stained with periodic acid-Schiff. The aorta tissue from descending aorta was cut, washed with 0.9% saline, and embedded in paraffin. After routine processing, paraffin sections of each tissue were cut into 4-μm thickness for hematoxylin-eosin (HE) staining and determination of collagen I.

### The detection of serologic indexes

The detection of Scr, UA, serum NO, serum ET-1, serum SOD, serum MDA, serum CRP, serum LDL, and ox-LDL was performed according to the instructions in the kits.

### Statistical analysis

The proportion of collagen I positive area was measured by randomly selecting three fields in each slide and dividing each field into 1,564 parts by Photoshop. The number of positive points were counted; the proportion was the number of positive points/1,564. Data were calculated by two examiners and the average values were calculated.

All data were expressed by x̄ ± s. Statistical analysis was performed using the Statistical Package for Social Sciences (SPSS for windows, version 13.5). Comparisons between groups were analyzed using the *t*-test. Variable comparisons were assessed using one-way analysis of variance (ANOVA) and multiple stepwise regression analysis. A *P* value < 0.05 was considered as significant.

## Results

### Early CKD animal model with hyperuricemia

Group A (sham operation) and group B (right nephrectomy only) served as controls. Group C (right nephrectomy with oxonate potassium) was the experimental group.

Periodic acid-Schiff staining of kidney tissues from each group showed mild glomerular mesangial proliferation in groups B and C, compared to group A (Figure 1A,C,E). No obvious pathological change in renal tubule and renal interstitium was visible in the three groups. Meanwhile, there was no renal tubular epithelial cells necrosis, no inflammatory cells in the interstitium, and no small vessel lesions in groups B and C (Figure 1D,F). In the experimental group, there was no urate crystal deposition. Compared with groups A and B, the experimental group had a significantly higher level of UA. However, there was no obvious difference in Scr among the three groups (Table 1), which was in accordance with the characteristics of early CKD. The above results indicate the establishment of an early CKD animal model with hyperuricemia.

The article "Effects of uric acid on endothelial dysfunction in early chronic kidney disease and its mechanisms" was retracted in 2015. Reasons: compromised peer review; ethical violations by an institution or third party; concerns about the results or conclusions.

**Figure 1:** **Pathological pictures of rat kidneys from groups A, B, and C. (A)** The normal renal glomerulus of group **A** (×400). **(B)** No obvious pathological change in renal tubules of group A (×400). **(C**, **E)** Mild glomerular mesangial proliferation in renal glomerulus of groups **B** and **C** (×400). **(D**, **F)** There were no obvious pathological changes in renal tubules in groups **B** and **C** (×400).

**Table 1:** **Concentration of Src, UA, P**_**CIPA**_**, NO, ET-1 and NO/ET-1 ratio in three groups (x̄±s)**

**Group**	**Scr (μmol/L)**	**UA (μmol/L)**	**P**_**CIPA **_**(%)**	**NO (μmol/L)**	**ET-1 (pg/mL)**	**NO/ET-1**
A	30.20 ± 6.01	53.10 ± 8.62	12.90 ± 2.31	47.55 ± 5.39	5.89 ± 1.67	8.18 ± 2.32
B	31.70 ± 4.72	53.70 ± 11.52	12.97 ± 2.71	45.34 ± 4.76	5.92 ± 1.56	8.90 ± 3.55
C	30.80 ± 5.90	161.40 ± 28.04^*^	22.38 ± 3.14^*^	36.71 ± 3.45^*^	7.50 ± 1.06^△^	5.07 ± 1.19^*^

Note:

^*^: *P* <0.01 group C vs. groups A and B.

^△^: *P* <0.05 group C vs. groups A and B.

P_CIPA_: Percentage of collagen I positive area.

### Vascular endothelial cell injury in the experimental group

In the light microscope, endothelial cells of group A were arranged closely under the vascular intima and inflammatory cells did not accumulate in the vascular wall (Figure 2A); smooth muscle cells were arranged in order with a spindle shape and an almost uniform morphology (Figure 2B). However, in group C, a foam-like interstitial edema of endothelial cells was visible (Figure 2E). Partial endothelial cells was shed from the vessel wall and the gap between them was broadened (Figure 2F). Further, inflammatory cells accumulated in the vascular intima (Figure 2G,H) and several inflammatory cells infiltrated within the membrane (Figure 2I,J). The thickness of the blood vessel wall increased. Medial smooth muscle cells proliferated and thickened with an irregular shape and a disordered arrangement (Figure 2K). The pathological change of the right-side nephrectomy group (group B) was similar to the experimental group, but less marked (Figure 2C). Smooth muscle cell proliferation was not obvious and it was well arranged (Figure 2D). The results confirmed significant vascular injury in the experimental group.

**Figure 2:** **Pathological images of rat arteries from groups A, B, and C. (A)** Endothelial cells arranged in order under the vascular intima of group **A** (×400). **(B)** There was no obvious proliferation of medial smooth muscle cells in the vascular wall of group **A** (×200). **(C)** The morphology of endothelial cells of group **B** was slightly abnormal (×400). **(D)** There was no obvious proliferation of medial smooth muscle cells in the vascular wall of group **B** (×200). **(E)** Endothelial cells of group **C** had a foam-like change (×400). **(F)** Endothelial cells of group **C** shed from the vessel wall (×400). **(G**, **H)** Inflammatory cells accumulated in the vascular intima of group **C** (×400). **(I)** Neutrophil granulocytes were seen around the endothelial cells of group **C** (×400). **(J)** Mononuclear cells were seen around the endothelial cells of group **C** (×400). **(K)** Smooth muscle cells of group **C** proliferated, thickened, and had no order (×200).

The article "Effects of uric acid on endothelial dysfunction in early chronic kidney disease and its mechanisms" was retracted in 2015. Reasons: compromised peer review; ethical violations by an institution or third party; concerns about the results or conclusions.

Collagen I staining of the vascular wall in the three groups is shown in Figure 3. Several collagen I depositions were visible in the vascular wall of groups A and B, while the collagen I component was significantly increased in group C. Statistical analysis showed that the percentage of collagen I positive area in the vessel wall of the experimental group was significantly higher than that of group A and group B (group C vs. group A, *P* < 0.01; group C vs. group B, *P* < 0.01) (Table 1).

**Figure 3:** **Collagen I staining of the vascular wall in groups A, B, and C. (A**,**B)** A small amount of collagen I deposition was seen in the vascular wall of group **A** (×400). **(C)** Collagen I component was significantly increased in group **C** (×400).

Blood NO and ET-1 were important values to reflect the function of endothelial cells. Compared to groups A and B, in the experimental group, serum NO level was low (*P* < 0.01), serum ET-1 level was high (*P* < 0.05), and the NO/ET-1 ratio was low (*P* < 0.01). The above results verified endothelial cell dysfunction and significant injury of vascular endothelial cells.

### Uric acid-induced vascular endothelial cell injury in early CKD

The possibility of a direct correlation between elevated UA level and vascular disease as well as endothelial injury was also investigated. Linear regression analysis showed that the level of serum UA had a significant positive correlation with the percentage of collagen I positive area (r = 0.8403, *P* < 0.01) and serum ET-1 (r = 0.9374, *P* < 0.01), but a negative correlation with serum NO (r = −0.9462, *P* < 0.01) and NO/ET-1 ratio (r = −0.9230, *P* < 0.01) (Table 2). The percentage of collagen I positive area had a significant positive correlation with serum ET-1 (r = 0.8737, *P* < 0.01), but a negative correlation with serum NO (r = −0.9171, *P* < 0.01) and NO/ET-1 ratio (r = −0.8707, *P* < 0.01) (Table 3). The results indicated that UA induced vascular endothelial cell injury in early CKD and the production of collagen I in the vascular wall. Meanwhile, the production of collagen I was relative to the injury of endothelial cells.

The article "Effects of uric acid on endothelial dysfunction in early chronic kidney disease and its mechanisms" was retracted in 2015. Reasons: compromised peer review; ethical violations by an institution or third party; concerns about the results or conclusions.

**Table 2:** **Correlation between serum uric acid and P**_**CIPA**_**, NO, ET-1, and NO/ET-1 ratio in the vascular wall**

	**Serum uric acid (μmol/L)**	
	**r value**	***P *value**
P_CIPA_ (%)	0.8403	0.0023
NO (μmol/L)	−0.9462	0.0000
ET-1 (pg/mL)	0.9374	0.0001
NO/ET-1 ratio	−0.9230	0.0001

**Table 3:** **Correlation between P**_**CIPA **_**in the vascular wall and NO, ET-1, and NO/ET-1 ratio**

	**P**_**CIPA **_**(%)**	
	**r value**	***P *value**
NO (μmol/L)	−0.9171	0.0002
ET-1 (pg/mL)	0.8737	0.0010
NO/ET-1 ratio	−0.8707	0.0010

### Uric acid caused vascular endothelial injury in early CKD by oxidative stress, micro-inflammation, and lipid oxidation mechanisms

The above experiments showed that UA was involved in early CKD vascular endothelial cell injury; however, the mechanism is unclear. Basic research demonstrated that UA crystals deposited in the intima could directly cause endothelial cell damage. Whether there are other important mechanisms apart from this remains to be investigated.

Our research showed that the experimental group had lower level of serum SOD (U/mL) compared with groups A and B (group C vs. group A, *P* < 0.01; group C vs. group B, *P* < 0.01) and higher level of serum MDA (nmol/mL) (group C vs. group A, *P* < 0.01; group C vs. group B, *P* < 0.05) (Table 4). Linear regression analysis showed that the level of serum UA had a significant positive correlation with serum MDA (r = 0.8195, *P* < 0.01), but a negative correlation with serum SOD (r = −0.6885, *P* < 0.05), which indicated that UA might lead to oxidative stress in early CKD. Further, the level of serum NO had a significant positive correlation with serum SOD (r = 0.8179, *P* < 0.01), but a negative correlation with serum MDA (r = −0.9171, *P* < 0.01). The level of serum ET-1 had a significant positive correlation with serum MDA (r = 0.8658, *P* < 0.01), but a negative correlation with serum SOD (r = −0.7793, *P* < 0.01). NO/ET-1 ratio had a significant positive correlation with serum SOD (r = 0.8143, *P* < 0.01), but a negative correlation with serum MDA (r = −0.9143, *P* < 0.01). SOD entered the multiple stepwise regression equation of NO and ET-1, indicating that oxidative stress can cause vascular endothelial dysfunction in early CKD (Table 5).

**Table 4:** Concentration of serum SOD, MDA, CRP, ox-LDL, and LDL in the three groups (x̄±s)

**Group**	**SOD**	**MDA**	**CRP**	**ox-LDL**	**LDL**
	**(U/mL)**	**(nmol/mL)**	**(μg/mL)**	**(mmol/L)**	**(mmol/L)**
A	249.80 ± 9.83	4.06 ± 0.28	10.43 ± 1.68	47.50 ± 11.51	0.18 ± 0.06
B	243.60 ± 8.11	4.04 ± 0.41	12.27 ± 2.76	53.31 ± 12.38	0.18 ± 0.06
C	224.40 ± 6.47^*#^	4.40 ± 0.23^△#^	14.68 ± 2.01^△#^	65.22 ± 10.91^△#^	0.25 ± 0.06^△#^

Note:

^*^: *P* <0.01 group C vs. group B.

^△^: *P* <0.05 group C vs. group B.

^#^: *P* <0.01 group C vs. group A.

The article "Effects of uric acid on endothelial dysfunction in early chronic kidney disease and its mechanisms" was retracted in 2015. Reasons: compromised peer review; ethical violations by an institution or third party; concerns about the results or conclusions.

**Table 5:** **Correlation between serum UA, NO, ET-1, and NO/ET-1 ratio as well as P**_**CIPA**_**, SOD, MDA, CRP, ox-LDL, and LDL**

	**Serum uric acid (μmol/L)**		**Serum NO (μmol/L)**		**Serum ET-1 (pg/mL)**		**NO/ET-1 ratio**		**P**_**CIPA **_**(%)**	
	**r value**	***P *value**	**r value**	***P *value**	**r value**	***P *value**	**r value**	***P *value**	**r value**	***P *value**
SOD (U/mL)	−0.6885	0.0277	0.8179	0.0038	−0.7793	0.0079	0.8143	0.0041	−0.8180	0.0000
MDA (nmol/mL)	0.8195	0.0037	−0.9171	0.0002	0.8658	0.0012	−0.9143	0.0002	0.8015	0.0053
CRP (μg/mL)	0.7251	0.0177	−0.7554	0.0115	0.7447	0.0135	−0.8042	0.0050	0.6752	0.0322
ox-LDL (mmol/L)	0.8479	0.0019	−0.7459	0.0132	0.7900	0.0065	−0.7949	0.0060	0.5266	0.1179
LDL (mmol/L)	0.6356	0.0483	−0.5080	0.1339	0.5734	0.0831	−0.4947	0.1460	0.5902	0.0725

Note: NO as dependent variable and SOD, MDA, CRP, ox-LDL, LDL as independent variables, multiple stepwise regression analysis showed that serum SOD and CRP entered the equation, and the equation was y = 0.315 × _1_-0.802 × _2_-22.120 (y = NO, ×_1_ = SOD, ×_2_ = CRP; -22.120 was a constant). ET-1 as dependent variable and SOD, MDA, CRP, ox-LDL, and LDL as independent variables, multiple stepwise regression analysis showed that serum ox-LDL and SOD entered the equation, and the equation was y = 0.051 × _1_-0.082 × _2_ + 22.517 (y = ET-1, ×_1_ = ox-LDL, ×_2_ = SOD; 22.517 was a constant). NO/ET-1 ratio as dependent variable and SOD, MDA, CRP, ox-LDL, LDL as independent variables, multiple stepwise regression analysis showed that serum SOD and CRP entered the equation, and the equation was y = 0.102 × _1_-0.316 × _2_-13.151 (y = NO/ET-1 ratio, ×_1_ = SOD, ×_2_ = CRP; 13.151 was a constant). P_CIPA_ as dependent variable and SOD, MDA, CRP, ox-LDL, LDL as independent variables, multiple stepwise regression analysis showed that serum SOD entered the equation, and the equation was y = 111.437-0.397 × _1_ (y = P_CIPA_, ×_1_ = SOD; 111.437 was a constant).

Our research also found that the experimental group had a higher level of serum CRP (μg/mL) compared with groups A and B (group C vs. group A, *P* < 0.01; group C vs. group B, *P* < 0.05) (Table 4), which indicated that the experimental group had a more obvious micro-inflammation state. Linear regression analysis showed that the level of serum UA had a significant positive correlation with serum CRP (r = 0.7251, *P* < 0.05), which indicated that UA was involved in the formation of micro-inflammation in early CKD. Further, the level of serum NO had a significant negative correlation with serum CRP (r = −0.7554, *P* < 0.05). Serum ET-1 level had a significant positive correlation with serum CRP (r = 0.7447, *P* < 0.05). NO/ET-1 ratio had a significant negative correlation with serum CRP (r = −0.8042, *P* < 0.01). CRP entered the multiple stepwise regression equation of NO and NO/ET-1 ratio, indicating that micro-inflammation was involved in the formation of vascular endothelial dysfunction in early CKD (Table 5).

The article "Effects of uric acid on endothelial dysfunction in early chronic kidney disease and its mechanisms" was retracted in 2015. Reasons: compromised peer review; ethical violations by an institution or third party; concerns about the results or conclusions.

By studying the levels of serum LDL and ox-LDL, we found that the experimental group had a higher level of serum LDL (mmol/L) than groups A and B (group C vs. group A, *P* < 0.01; group C vs. group B, *P* < 0.05) and a higher level of serum ox-LDL (mmol/L) (group C vs. group B, *P* < 0.05) (Table 4). Linear regression analysis showed that the level of serum UA had a significant positive correlation with serum ox-LDL (r = 0.8479, *P* < 0.01) and serum LDL (r = 0.6356, *P* < 0.05), which indicated that UA can cause lipid metabolic disorder in early CKD. Further, the level of serum NO had a significant negative correlation with serum ox-LDL (r = −0.7459, *P* < 0.05), but no significant correlation with serum LDL (r = −0.5080, *P* > 0.05). Serum ET-1 levels had a significant positive correlation with serum ox-LDL (r = 0.7900, *P* < 0.01), but no significant correlation with serum LDL (r = 0.5734, *P* > 0.05). NO/ET-1 ratio had a significant negative correlation with serum ox-LDL (r = −0.7949, *P* < 0.01), but no significant correlation with serum LDL (r = −0.4947, *P* > 0.05). Serum ox-LDL entered the multiple stepwise regression equation of ET-1 (Table 5). The results indicated that ox-LDL had strong endothelial cell toxicity.

In addition, the percentage of collagen I positive area in the vascular wall had significant positive correlations with serum MDA (r = 0.8015, *P* < 0.01) and serum CRP (r = 0.6752, *P* < 0.05), a negative correlation with serum SOD (r = −0.8180, *P* < 0.01), and no significant correlation with serum ox-LDL (r = 0.5266, *P* > 0.05) or serum LDL (r = 0.5902, *P* > 0.05) (Table 5). Multiple stepwise regression analysis showed that serum SOD entered the equation. According to the results, it was found that oxidative stress and micro-inflammation could lead to an increase of collagen I deposition in the vessel wall. However, whether lipid metabolism disorders had a relation with increased collagen deposition in the vessel wall was not determined.

The article "Effects of uric acid on endothelial dysfunction in early chronic kidney disease and its mechanisms" was retracted in 2015. Reasons: compromised peer review; ethical violations by an institution or third party; concerns about the results or conclusions.

In conclusion, UA caused endothelial dysfunction in early CKD via mechanisms involved in oxidative stress, micro-inflammation, and abnormal lipid metabolism.

## Discussion

In this study, serum UA levels in rats were elevated with potassium oxonate by gavage. In 1965, it was verified that potassium oxonate had a strong ability to inhibit uricase activity both *in vivo* an *in vitro*[17]. Many reports have established a hyperuricemia animal model with potassium oxonate [18]. In this study, we compared the morphology and biochemical changes of kidney cells between the experimental group and the control group, as well as a unilateral nephrectomy group. The experimental group and the unilateral nephrectomy group had no obvious glomerular lesions; only some of the glomerulus presented mild mesangial proliferation. No obvious abnormality of renal tubules and renal interstitium was visible. Meanwhile, hyperuricemia kidney disease caused by urate crystal deposition was not visible in the experimental group. In serology, serum creatinine levels among the three groups had no significant difference (*P* > 0.05). Nevertheless, the serum UA level of the experimental group was significantly higher than the other two groups (about three times). Therefore, we believe that an early-CKD animal model with hyperuricemia was successfully established.

Endothelial dysfunction is prevalent in CKD patients, and in particular end-stage renal disease patients [19]. Many factors lead to endothelial dysfunction, the mechanisms of which have not been clearly elucidated as yet. Because of abnormal changes in UA excretion through the kidney, serum UA levels are higher in CKD patients compared to the normal population and serum UA continues to rise with deterioration of renal function. Many researchers reported that UA was elevated in CKD and might play a role in the pathophysiology of CKD progression through endothelial dysfunction, such as activation of local renin-angiotensin system, increased oxidative stress, and proinflammatory and proliferative actions [20-22]. This conclusion, although controversial, was supported in *in vitro* experimental studies showing the relationship of UA with NO production and depletion [23,24]. Given that contention, it was necessary to study the relationship of UA with early CKD vascular endothelial injury through animal experiments.

Our experiment showed that the endothelial cells of the experimental rats presented obvious morphological changes. In normal circumstances, vascular endothelial cells inhibit inflammatory cell adhesion and anti-smooth muscle cell proliferation and migration. However, in experimental rats, aggregation of inflammatory cells was observed in the vessel wall, which was even infiltrated into the intima, accompanied by vascular wall was thickening. Further, smooth muscle cells were hyperplastic, thickened, irregular, and disorganized. In addition, immunohistochemical methods demonstrated that collagen I increased significantly in the vessel wall. Hence, the above vasculopathy can be regarded as a consequence of endothelial injury.

The article "Effects of uric acid on endothelial dysfunction in early chronic kidney disease and its mechanisms" was retracted in 2015. Reasons: compromised peer review; ethical violations by an institution or third party; concerns about the results or conclusions.

Endothelial cells, an important endocrine organ, can secret many important active substances that play important roles in the cardiovascular system, such as NO, prostacyclin hormone, endothelin, angiotensin, antithrombin III, and plasminogen activator. These substances are useful for homeostasis in the normal case; when the homeostasis balance is broken, the secretion is abnormal. Therefore, to a certain extent, endothelial cell function can be assessed by detecting the concentration of these substances in the serum. In our study, the substances of contraction and relaxation of vascular NO and ET-1 [25], synthesized and secreted by endothelial cells respectively, were used to assess endothelial cell function. The study found that serum NO concentration of the experimental group was significantly low and ET-1 was significantly high compared to the unilateral nephrectomy group, indicating that NO and ET-1 secretion were out of balance. Therefore, we believe that there is a significant endothelial dysfunction in the experimental group. Further, line correlation analysis showed that serum UA level was significantly correlated with the endothelial function indicators NO and ET-1, indicating that UA has a relation to vascular endothelial cell dysfunction and participates in early CKD vascular endothelial cell injury.

Increased oxidative stress and reduced antioxidant capacity are prevalent in CKD patients [26]. Even in patients with mild renal impairment, oxidative stress level has increased more significantly than the normal population. The level of oxidative stress will intensify as renal deterioration. Oxidative stress plays an important role in endothelial cell damage and functional changes [27]. At present, studies on oxidative stress and endothelial injury mainly focus on end-stage renal disease patients [28]. The present study focuses on early CKD, and found that the experimental group has a significant increased oxidative stress level related to serum UA concentration, indicating that UA is involved in the formation of the early CKD oxidative stress status.

Systemic micro-inflammation is widespread in CKD patients, even accompanied by mild renal dysfunction [29]. At present, the degree of inflammatory response is closely related to the incidence and mortality of cardiovascular events in CKD patients [30,31]. CRP is an acute phase protein synthetized by liver in inflammation, which is recognized as a reliable marker reflecting the inflammatory state. Our study found that the CRP level of the experimental group was significantly higher than the unilateral nephrectomy group, indicating that the micro-inflammatory state of the experimental group was more obvious. CRP level was significantly correlated with serum UA level, showing that UA is involved in the formation of micro-inflammation in early CKD. Further analysis showed that serum CRP level was significant correlated with NO, ET-1, and NO/ET-1 ratio, all of which are indicators of endothelial function. CRP entered the NO and ET-1 multiple regression equation, indicating that micro-inflammation is involved in vascular endothelial cell damage of in early CKD.

The article "Effects of uric acid on endothelial dysfunction in early chronic kidney disease and its mechanisms" was retracted in 2015. Reasons: compromised peer review; ethical violations by an institution or third party; concerns about the results or conclusions.

CKD is often accompanied by lipid metabolic disorders, including increased plasma lipoprotein concentrations and/or lipoprotein composition changes [32]. Our study found that in the experimental group LDL levels, as well as its oxidized form ox-LDL, were increased compared to the unilateral nephrectomy group, both of which were significantly correlated with UA, suggesting that UA leads to early CKD lipid metabolic disorders. Further analysis showed that LDL was not significantly correlated with endothelial function indicators NO and ET-1, but its oxidized form was significantly associated with these indicators. Lipid metabolism disorders might be involved in endothelial cell damage. It is believable that only ox-LDL has strong endothelial cell toxicity compared to LDL. The higher the degree of oxidation, the stronger the damage is. Our findings also confirmed this.

Finally, a correlation study about the percentage of collagen I positive area of the vessel wall and serum UA levels, endothelial function indicators NO, ET-1, and NO/ET-1 ratio, as well as the activities of SOD, MDA, CRP, LDL, and ox-LDL indicated that the percentage of collagen I positive area of the vessel wall was significantly associated with serum UA level, NO, ET-1, NO/ET-1 ratio, SOD, MDA, and CRP, but had no obvious correlation with LDL and ox-LDL. Based on the above, we believe that UA causes vascular endothelial cell injury in early CKD and leads to collagen proliferation in the vessel wall. Meanwhile, collagen hyperplasia has a relation to endothelial cell injury. We found that oxidative stress and micro-inflammation can lead to increased collagen I deposition in the vessel wall, but whether lipid metabolism disorders are associated with increased collagen component deposition in the vessel wall is not yet determined. With the percentage of collagen I positive area as a dependent variable, multiple stepwise regression analysis showed that serum SOD entered the equation. Based on these results, we speculate that micro-inflammation can lead to collagen I proliferation, but oxidative stress may act in the final passage leading to increased collagen deposition in the vessel wall.

The article "Effects of uric acid on endothelial dysfunction in early chronic kidney disease and its mechanisms" was retracted in 2015. Reasons: compromised peer review; ethical violations by an institution or third party; concerns about the results or conclusions.

## Conclusions

In summary, this study successfully established an early-CKD animal model with elevated serum UA by unilateral nephrectomy plus potassium oxonate intragastrically. With the animal model, we found UA had a role in early CKD vascular endothelial cell injury. UA is involved in the formation of oxidative stress, micro-inflammatory state, and abnormal lipid metabolism in early CKD, based on which UA may lead to early CKD vascular endothelial injury. Therefore, strengthened control the UA level in early CKD aiming to correct oxidative stress, micro-inflammatory state, and lipid metabolism disorders, could improve vascular endothelial function, delay the process of atherosclerosis, and improve quality of life for CKD patients.

## Abbreviations

CKD: Chronic kidney disease; CRP: C-reactive protein; CVD: Cardiovascular disease; ET-1: Endothelin-1; LDL: Low density lipoprotein; MDA: Malonaldehyde; NO: Nitric oxide; ox-LDL: Oxidatively modified low-density lipoprotein; Scr: Serum creatinine; SOD: Super oxide dismutase; TGF-β: Transforming growth factor-β; UA: Uric acid.

## Competing interests

The authors declare that they have no competing interests.

## Authors’ contributions

YW: Designed the experiments, and acquired and analyzed the data. XRB: Designed the experiments and drafted the manuscript. Both authors read and approved the final manuscript.
